The article "Optimization of Online Course Platform for Piano Preschool Education Based on Internet Cloud Computing System" was retracted in 2023. Reasons: unreliable results or conclusions; lack of ethics approval or compliance; concerns about the data; concerns about the peer review.

# Optimization of Online Course Platform for Piano Preschool Education Based on Internet Cloud Computing System

**DOI:** 10.1155/2022/6525866

**Published:** 2022-06-15

**Authors:** Qianru Hu

**Affiliations:** School of Educational Sciences, Guangxi Science and Technology Normal University, Laibin, Guangxi, 546199, China

## Abstract

This article focuses on introducing online piano teaching methods and has developed and implemented a preschool piano education online course platform. The system consists of four parts: backend, WeChat, client, and web page. Backend development uses PHP language and Laravel system framework, WeChat and web development both use JavaScript language and React framework, client development uses Objective-C language, and the system provides internal support for RESTful API, mainly for client, WeChat, and web. The client relies on the existing voice sensors of the research group to recognize and evaluate the performance of the students. The role of the client is to show the students their homework and demonstrate the activities performed by the teacher. The function of the WeChat terminal is to manage student work, user information, and user social interaction functions. The function of the web page is the score management and data analysis functions. Based on the knowledge of network course design, this article studies the design of piano preschool education platform and adds relevant components of the Internet cloud computer system and voice sensor to this platform, which provides great convenience for students to learn piano.

## 1. Introduction

The rapid development of the Internet makes online education more and more developed [1]. At this stage, most online education is done through videos of traditional courses, and Internet education is currently indispensable. In terms of quality education, especially in the field of music education, many companies and institutions have begun to develop intelligent online music education products in order to improve the effectiveness of teacher teaching and the learning effect of students [2]. Based on the above analysis and research, this article aims to use the Internet cloud computing system and sound sensors to create an online piano preschool education course platform to solve the challenges of traditional piano preschool education so that teachers or parents can assign online homework to students [3]. Students can use the online course platform to practice piano at home. The online course platform can provide real-time evaluation, which can let students know the results of their practice and correct them in time if there are errors [4]. At the same time, parents and teachers can follow their children's learning achievements online in real time and improve their teaching results [5]. The system has passed extensive performance tests and functional tests, and the current system architecture is stable and reliable enough to meet current needs [6]. This article introduces the needs, analysis, design, application, and testing of the preschool piano education online course website. The system can provide greater convenience and better teaching results for traditional preschool piano teaching and help students learn piano from parents and teachers [7]. It provides tools for supervising and managing piano learning and enables teachers, parents, and students to communicate smoothly, quickly, and without barriers based on voice sensors. Now, the system has been connected to the Internet. At present, 27 books have been registered, 1,257 electronic music score resources, 6,714 recording data materials, and 753 registered users. The system has been widely praised by consumers. At the same time, from the feedback information, the system is constantly updated and improved to achieve better service effects.

## 2. Related Work

The literature is based on the piano accompaniment of the smart camera, which integrates the smart system and the traditional teaching system, and its purpose is to achieve better teaching effects [8]. On the iPad APP, teachers can pay attention to the piano keyboard area where students are learning in real time and provide real-time guidance and teaching. In the teaching application, teachers can mark pages of scores and synchronize student notes, just like in one-to-one teaching [9]. At the same time, this auxiliary teaching program uses a piano performance evaluation method based on artificial intelligence technology, which can evaluate the pitch and speed of students' performance in real time [10]. And this teaching plan classifies the courses to meet the learning needs of students of different ages. The document design realizes the application of the WeChat official account, which can enable parents to learn about students' information, can assist parents and teachers in supervising and managing students' learning conditions, and can also assist the principal in managing teacher information [11]. When setting up the WeChat official account application, it should be simple and easy to use, providing good use effects for students, parents, teachers, and principals. The literature designs and implements a client application that uses the existing multitone detection algorithm of the research team to help students view and complete assignments and can assist teachers with demonstration courses [12]. The client application plays the teacher's demonstration performance and pays attention to and evaluates the performance of the students in real time so as to solve the mistakes of the students practicing the piano without guidance. The literature introduces the research background of the art training management system and the importance of the current project research, and on this basis, uses a structured analysis method to investigate and analyze its main needs [13]. The literature draws a data flow diagram related to each process, classifies the general functional structure of the system and the structure of each functional module; in the data analysis stage, this article analyzes the data that each computer function needs to process and gives each organizational attribute chart of the organization.

## 3. Internet Cloud Computing System and Voice Sensor Technology

### 3.1. Internet Cloud Computing System

When users use cloud resources to perform computing tasks, they must send their own task requests to the server cluster on the local computer, and multiple computer resources in the cloud will work in response to the user's request and send the result decision to the local user, simplifying the user's local development process.

As cloud computing changes its computing methods, users' perception of using computer resources has changed from “purchasing materials” to “purchasing services.” In the traditional computer model, users buy real hardware or utility software. In addition to the direct cost of purchasing the product, users must also pay more to create a computer environment. In the context of cloud computing, users do not have to deal with complex hardware and software. They only need to spend a certain fee to enjoy the required services; users can achieve the purpose of purchase according to the requirements, avoiding losses caused by the loss of passive resources.

Compared with traditional computing models, cloud computing has the following characteristics:

1. High economy: users do not need to deploy clusters, saving hardware purchase and maintenance costs and paying as needed to avoid economic losses caused by the loss of passive resources.
2. Scalability: due to the gradual maturity of virtualization technology, most of the software and hardware resources have certain support for virtualization, so different resources can be added to the cloud computing cluster.

The cloud computing platform is a huge resource network, which integrates a large number of computer resources and provides computer services to external parties through the network. Its structure is shown in Figure 1.

  User layer: it is the entrance for users to access the cloud computing platform. Generally used for the user to send service requests and the user to communicate with the server function.
  Service list: after obtaining the permission, the user can access the cloud computing system and view the service list of the cloud computing system.
  System management and implementation tools: this module is responsible for managing users and managing computing resources.
  Resource tracking: this module is mainly used to monitor the usage of computer resources in the cloud computing system.
  Service cluster: a background cluster used to perform computing tasks and execute user requests.

In the computer system, communication can be carried out between nearby CUs. After the mobile terminal owned by the user enters the computer, it wirelessly connects to the nearest computing unit and sends a computing request to the computing unit.

(1) $$\begin{array}{c} S_{cp}=\frac{S_{cu}}{K}. \end{array}$$

### 3.2. Voice Sensor Technology

Suppose the light intensities of two monochromatic lights with the same frequency are I_1_ and I_2_, and their complex amplitudes are as follows:

(2) $$\begin{array}{c} E_{1}=I_{1}^{1/2}\cdot e^{i\phi_{1}},\\ E_{2}=I_{2}^{1/2}\cdot e^{i\phi_{2}}. \end{array}$$

Then the complex amplitude of the composite wave is as follows:

(3) $$\begin{array}{c} E=E_{1}+E_{2}. \end{array}$$

The light intensity of the synthesized wave is as follows:

(4) $$\begin{array}{c} I={\left|E\right|}^{2}={\left|E_{1}+E_{2}\right|}^{2},\\ ={\left|E_{1}\right|}^{2}+{\left|E_{2}\right|}^{2}+E_{1}^{*}\cdot E_{2}+E_{1}\cdot E_{2}^{*}, \end{array}$$

which is

(5) $$\begin{array}{c} I=I_{1}+I_{2}+2\cdot \sqrt{I_{1}\cdot I_{2}}\cdot \text{cos}\left(\phi_{1}-\phi_{2}\right). \end{array}$$

*k* represents the wave number of the laser light wave, *n* represents the refractive index of the fiber core, and the phase shift produced by the laser light wave through a length of *L* fiber is as follows:

(6) $$\begin{array}{c} \phi =k\cdot n\cdot L=\beta \cdot L. \end{array}$$

Differentiate equation (6) to get the following:

(7) $$\begin{array}{c} \Delta \phi =\Delta \left(\beta \cdot L\right),\\ =\beta \cdot L\cdot \varepsilon +L\cdot \frac{\partial \beta }{\partial n}\cdot \Delta n+L\cdot \frac{\partial \beta }{\partial a}\cdot \Delta a. \end{array}$$

Among them, the Poisson effect has a smaller influence on the phase of light waves than the other two factors, so calculations are not necessary. Since *β* = *n*•k,

(8) $$\begin{array}{c} \frac{\partial \beta }{\partial n}=\frac{\partial \left(n\cdot k\right)}{\partial n}=k. \end{array}$$

To simplify, formula (9) can be written as follows:

(9) $$\begin{array}{c} \Delta \phi =\Delta \phi_{1}+\Delta \phi_{2}. \end{array}$$

According to the strain theory, the normal strain vector of the optical fiber under the action of the stress *P* can be obtained:

(10) $$\begin{array}{c} \varepsilon =\left[\begin{array}{c} \varepsilon_{x}\\ \varepsilon_{y}\\ \varepsilon_{z} \end{array}\right]=\left[\begin{array}{c} \frac{-P\left(1-2\mu \right)}{E}\\ \frac{-P\left(1-2\mu \right)}{E}\\ \frac{-P\left(1-2\mu \right)}{E} \end{array}\right]. \end{array}$$

In the formula, *E* is Young's modulus of the optical fiber material, and Ʋ is Poisson's ratio of the optical fiber material. Since light waves propagate in the *z*-direction in the fiber, only the *z*-direction is considered; then,

(11) $$\begin{array}{c} \Delta \phi_{1}=\beta \cdot L\cdot \varepsilon_{z}=\frac{-\beta \cdot L\cdot P\left(1-2\mu \right)}{E}. \end{array}$$

According to the bounce effect, there are

(12) $$\begin{array}{c} \Delta \left(\frac{1}{n^{2}}\right)=\sum_{i=1}^{6}p_{ij}\cdot \varepsilon_{j}. \end{array}$$

When a uniform pressure is applied to the sensitive fiber, no shear stress will be generated, and the three main strains have the same effect on the upper pressure.

So there are only *j* = 1,2,3 components, at this time:

(13) $$\begin{array}{c} p_{ij}=\left[\begin{array}{ccc} p_{11} & p_{12} & p_{12}\\ p_{12} & p_{11} & p_{12}\\ p_{12} & p_{12} & p_{11} \end{array}\right]. \end{array}$$

From this, we can get the following:

(14) $$\begin{array}{c} \Delta {\left(\frac{1}{n^{2}}\right)}_{x,y,z}=p_{11}\varepsilon_{x}+p_{12}\varepsilon_{y}+p_{12}\varepsilon_{z},\\ =\frac{-\left(1-2\mu \right)\left(p_{11}+2p_{12}\right)}{E}\cdot P. \end{array}$$

Since the light wave propagates in the *z*-direction, it only affects the *x *- and *y-*directions, so

(15) $$\begin{array}{c} \Delta n\approx -\frac{2}{n^{3}}\Delta \left(\frac{1}{n^{2}}\right). \end{array}$$

But

(16) $$\begin{array}{c} \Delta \phi_{2}=k\cdot L\cdot \Delta n,\\ =\frac{2kL\cdot \left(1-2\mu \right)\left(p_{11}+2p_{12}\right)}{n^{3}\cdot E}\cdot P. \end{array}$$

Therefore, when the stress *P* acts on the optical fiber of length *L*, the phase change of the light wave propagating in the optical fiber is as follows:

(17) $$\begin{array}{c} \Delta \phi =\Delta \phi_{1}+\Delta \phi_{2},\\ =\frac{\beta \cdot L\cdot \left(1-2\mu \right)}{E}\cdot \left[\frac{n^{2}\cdot \left(p_{11}+2p_{12}\right)}{2}-1\right]\cdot P=\zeta \cdot P. \end{array}$$

The light wave propagating in the Sagnac interference ring is a physical quantity that changes with space and time. Considering that the optical fiber is an excellent linear medium, the light wave propagating clockwise in the interference ring can be expressed as follows:

(18) $$\begin{array}{c} E\left(x,y,z,t\right)=E_{s}\left(x,y,z\right)\cdot e^{i\omega t}. \end{array}$$

Among them, *x*, y, and *z* are three orthogonal directions in space, *t* represents the propagation time of the light wave, and *w* is the angular frequency of the light wave. The process of light propagation in a linear medium satisfies the following:

(19) $$\begin{array}{c} \nabla^{2}\cdot E\left(x,y,z,t\right)-\frac{n^{2}}{c^{2}}\cdot \frac{\partial^{2}E\left(x,y,z,t\right)}{\partial t^{2}}=0, \end{array}$$

which is

(20) $$\begin{array}{c} \nabla^{2}\cdot E_{s}\left(x,y,z\right)+\frac{n^{2}\cdot \omega^{2}}{c^{2}}\cdot E_{s}\left(x,y,z\right)=0. \end{array}$$

The light wave propagating in the counterclockwise direction in the Sagnac interference ring can be written as follows:

(21) $$\begin{array}{c} E^{\prime }\left(x,y,z,t\right)=E_{s}\left(x,y,z\right)\cdot e^{-i\omega t}. \end{array}$$

Due to the delayed rotation, the light wave in the Sagnac fiber interferometer has a different analysis time, which is different from the clockwise and counterclockwise connections. The time difference can be expressed as follows:

(22) $$\begin{array}{c} T_{\text{delay}}=\frac{n\left(L_{cc}-L_{c}\right)}{c}. \end{array}$$

When voice vibration acts on the probe, at time *t*, the phase difference between the two light waves can be expressed as follows:

(23) $$\begin{array}{c} \Delta \phi \left(t\right)=\Delta \phi \left(t-T_{\text{delay}}\right)-\Delta \phi \left(t\right). \end{array}$$

Suppose the pressure change caused by voice vibration is as follows:

(24) $$\begin{array}{c} \Delta P=P_{s}\text{cos}\left(\omega_{s}t\right). \end{array}$$

Combining formulas (22)–(24), the following can be obtained:

(25) $$\begin{array}{c} \Delta \phi \left(t\right)=2\cdot \zeta \cdot P_{s}\cdot \text{sin}\frac{\omega_{s}T_{\text{delay}}}{2}\cdot \text{sin}\left(\omega_{s}t-\frac{\omega_{s}T_{\text{delay}}}{2}\right). \end{array}$$

### 3.3. Simulation Analysis

According to the simulation parameters, the simulation results are shown in Figure 2. The horizontal axis in the figure is intensity, that is, the number of users entering the system per second, and the vertical axis represents the average waiting time for computing requests, not counting processing time. In the simulation, the time interval is set to 1 ms, so the vertical axis is represented by time, but the actual result is not related to the time slot size.

In Figure 3, the ideal situation is that after each user logs in to the system, the system allocates the idlest CU processing. Looking at the curve in the image, some conclusions can be drawn that the system is in a stable state before the intensity of 250 users/sec. The average waiting time interval obtained by the meter operating system is the smallest, and the simulation result is the best. The gap between the two varies with intensity.

## 4. Piano Preschool Education Network Course Platform Design and Optimization Research

### 4.1. Platform Demand Analysis

For online piano preschool education websites, the analysis of system requirements is definitely inseparable from students. The online course platform for piano preschool education in this article is for children under 5 years old, so parents' participation is needed to get good teaching results. At the same time, in order to establish a good relationship with the organization, teacher participation is essential, and it is also necessary to manage teachers through the principal.

Through the above analysis of the overall needs of computers, the target groups of users of the preschool piano education online course website are roughly divided into five categories: computer administrators, parents, students, teachers, and principals. The following will analyze the operational needs of these five consumer groups.

#### 4.1.1. Analysis of Administrator Functional Requirements

The administrator is the person who manages the piano preschool education network course platform, uploads and manages music scores through the computer, views and analyzes the performance data of students, and analyzes their user behavior.

*(1) Book Upload and Management*. After logging in to the system, you must first add specific piano books. Each list has the cover and title of the piano book, so it is easy to find the track you are looking for, and the administrator can edit and delete the uploaded book.

*(2) Upload and Manage Music Scores*. Administrators can click to enter the book to view a list of all electronic music scores in the book. Staff can edit and manage this information, such as title, English name, cover, and number of pages in a book. When there are too many scores, you can also display them in pages.

*(3) View and Analyze Performance Data*. To view the performance data list, the administrator should click Performance Data Analysis. Each part of the performance data includes the producer of the data, the performance time, and the performance score. The data analyzed by the administrator algorithm can be downloaded by clicking the download button. When there is too much data, a pagination display is also supported.

*(4) Analyze User Behavior*. Administrators can click Analyze to view a list of user behaviors. At the same time, the system supports filtering logs and user nickname search functions.

#### 4.1.2. Analysis of Parents' Functional Needs

Parents are the administrators responsible for managing students and the hub for communication with teachers. They hope to use this system to assign homework, view homework, manage students, and connect teachers and students.

*(1) View Homework*. Parents can view the homework assigned by the teacher and the homework assigned by the parent, as well as the homework completed by the student, and check the completion and quality of the homework.

*(2) Manage Students, Parents, and Teachers*. Parents can add a student, edit student information, and view the student's total practice time and frequency. At the same time, parents can bind another parent of a student with the system so that the bound parent can also see the student's homework and performance information.

#### 4.1.3. Analysis of Students' Functional Needs

The main requirement of the piano preschool education course website for students is to complete homework and check the performance. It is hoped that the system can strengthen the practice of skills and improve the quality of contact, while communicating with students from all over the world.

*(1) Complete Homework*. For online learning sites for piano education, letting students play is a very important requirement. When a student starts to play, the system will automatically call the tracked score and recognize the quality of the student's performance.

*(2) Check Out the Performance*. Preschool piano education online courses for toddlers not only meet the training needs of students but also meet the listening needs of students. For the music score, students should check the demonstration performance of this music score. The demonstration performance is produced by the teacher and can be watched when the teacher and students are bound. In addition, students should check the music they play to improve their learning level. Students can also check the performance of other students and understand the performance of other students.

#### 4.1.4. Analysis of Teachers' Functional Needs

Teachers teach offline piano to one or more people at a time and use the online piano preschool education network to provide students with homework, check homework, demonstrate to students, and supervise student training and teaching.

*(1) Assign and Check Homework*. After the teacher finishes teaching the students, they often ask the students to practice the content of the class after class. Teachers can choose the number of exercises on the piano preschool education course platform and assign relevant scores and homework to students. At the same time, the teacher should check the performance of each student and the completion of homework on the computer.

*(2) Performance Demonstration.* When students practice after class, similar demonstrations are often held. Teachers demonstrate through piano preschool education network courses to enhance the sense of teaching experience and teaching results.

#### 4.1.5. Analysis of the Principal's Functional Requirements

The principal is the coordinator of the online course platform for piano preschool education, hoping to coordinate the management of the entire school through this system.

*(1) Teacher Development.* The principal needs to bind the teacher to the school so that all students associated with the teacher will join the school.

### 4.2. Platform Function Design

Based on the analysis of computer requirements, this article divides the piano preschool education online course website into three parts: client, WeChat, and web. The function modules of the system function design shown in Figure 4 are described in detail below.

#### 4.2.1. Client Function Design

*(1) Square Module*. The square module is mainly responsible for the communication function between teachers and students. The current users who are currently logged in at the same school and the same teacher will present the users concerned in the form of cards. The cover is the user's avatar, the latest song can be displayed under the card, and then click on the card to enter the next level page, the user information in the next level page is displayed on the left, the playing card is displayed on the right, and the playing time is arranged in reverse order.

When the user is a teacher, click on the card to enter the demonstration teaching. The teacher can add demonstration exercises by himself, and the teacher can click the demonstration performance to start playing. Here the teacher has a correction function, the teacher can mark the errors and difficulties that appear on the system, and then the marked notes and the dragged scores are stored in the system file. When students play this piece, they can use this demonstration video to practice, and students can click to download and play back to learn.

#### 4.2.2. WeChat Terminal Function Design

*(1) User Management Module*. The user management module includes functions such as user registration, user information modification, and user binding. When the user clicks on the student menu, the server first receives the user's WeChat openid and then queries the MySQL server to verify whether the user is on the parent table of the MySQL database.

Parents can edit their personal information or children's information using the avatar name, avatar, background picture, piano age, and name and can also add and delete information.

There are three types of user binding: one is the teacher binding the principal, the other is the parent adding a teacher to the child, and the third is the parent adding a teacher. When the principal clicks on Teacher Development, a QR code will appear at the top of the page, and a list of school teachers will appear at the bottom of the page. Teachers can scan the WeChat QR code provided by the principal to bind with the school. After binding, the teacher can create a unique class number, and the parent can add a teacher for the child by clicking the add button and entering the class number.

*(2) Job Module*. The job module is composed of two parts: job layout and job viewing. Students' homework can be assigned by teachers or parents.

The teacher clicks on the student card to enter the homework view. The homework view is displayed by cards. There are three types of cards. The first card is the teacher assigning homework to the students. The card information includes the name of the teacher, the name of the student, the assigned time, and the number of tracks. If the student has practiced the repertoire, the information also includes the start time, practice time, and the number of stars obtained this time during the training. The second type of card is used by parents to assign homework to the student, which is similar to the card used by the teacher to assign homework to the student, but the teacher's name is changed to the parent's name. The third card is the computer system information, which contains the welcome message for the user to use the piano online course for the first time and the information on the student's score. Click on the student's score to view the list of all recordings.

### 4.3. Database Design

Piano preschool education online courses cover a lot of entity objects, and the relationship between the objects is relatively strong, so we choose a MySQL database that supports a relatively good relationship to create the database that the computer needs. For the database server, we chose Alibaba Cloud's MySQL database server to support our business.

The parent table is used to store the personal information of the parent. The specific fields of the parent table are shown in Table 1.

The student table is mainly used to store the personal information of students created by parents. The specific fields of the student table are shown in Table 2.

This table is used to store the binding relationship between parents and families. The specific fields of the parent_family_relationship table are shown in Table 3.

The opern table is used to store the basic information of the score. The specific fields of the opern table are shown in Table 4.

The record information is stored in the recording table, which not only stores the information related to the student's training record but also stores the information related to the type of individual teacher's performance record by field type. The specific fields of the recording table are shown in Table 5.

### 4.4. Platform Process Optimization

The piano preschool education online learning website uses a traditional manual management system, but under the manual management system, the personnel management ability is low, which decentralizes the decision-making to a certain extent and affects the efficiency of its decision-making, so the original business process must be carried out for optimization and improvement.

Reimproving the original business process, taking into account the development of the art center's own organizational structure and the introduction of modern computer technology, the main problem is to reorganize the core business process to meet actual business needs and scientifically and effectively handle the flow of data content, which is suitable for the business management process of system design and is also the purpose of our system optimization.

Compared with the traditional process, the registration and registration optimization process can be completed by reviewing basic student information, finding old student files, installing new student files, and opening selected courses. It enables employees to reduce their workload and put more energy into education management. Because the formatting of data is done by a computer system, the chance of formatting errors is almost zero.

According to financial statistics, the traditional method is to collect all the application forms and then manually calculate the number of applicants and total fees for the semester, which is not only a lot of work but also prone to errors. However, in the customized process, all the work is managed by the system, and only the financial staff will automatically prepare the financial statements when the registration deadline is reached. Data acquisition, personnel statistics, and charging status are all completed by the system.

Because the system management reduces the human intervention in the charging process, the error rate of human financial problems is greatly reduced, the safety of funds is very effectively guaranteed, and the occurrence of financial loopholes is avoided.

### 4.5. Teaching Analysis and Development

*(1) Feasibility Analysis*. It mainly depends on whether the online teaching website of Moodle can realize the teaching effect of combining designer classroom teaching and offline network teaching. Enough data and tests are used to prove the feasibility of this teaching process and whether it is financially and technically feasible. Detailed evaluation and analysis are shown in Figure 5. The biggest advantage of this framework is that it can be used anywhere as long as it can be connected to the Internet, and it has very strong operability.

The design policy should be consistent with the learner's knowledge level and should not exceed the learner's knowledge and skills. Design and development include the following functions.

Teaching content design is a very important part of teaching. A large number of learning resources are the source of knowledge for learners. When designing curriculum resources, we should carefully consider the ability to accept the information materials, the impact of the materials on students and whether they are suitable, the development of students, and the knowledge that students need.

Constructivist teaching system design focuses on learning in a learning context, provides students with real-time learning methods, restores the richness and vividness of knowledge, takes teaching as the starting point, lets students participate in learning more actively, and establishes practical knowledge definitions.

Independent learning strategies are used to stimulate students' initiative and enthusiasm. Teaching strategies include preclass activities, information transmission, reasonable use of teaching media, and the combination of classroom teaching and online teaching. Then interactive teaching results are produced, the teaching process fully reflects the “student” as the main organization, and comprehensive teaching content needs to be presented in different ways, at different times and in different environments. Also, consider subjective factors, objective factors ,and social factors, and choose different learning strategies.

## 5. Conclusion

Today's society is a society where online education is popular and information is updated rapidly. The network resources are relatively rich, and the Internet cloud computing system is used as a platform to provide new tools for the expansion and communication of preschool children's education. As a parent, you can watch the children's performance in the kindergarten and contact the teacher for feedback in time; as a child, you can learn more and more interesting knowledge from the platform; as a teacher, you can have more exchanges and learn about each. The child's situation allows every child to be paid attention to and then to be taught in accordance with their aptitude. According to the needs of the subject, based on the voice sensor combined with the current pain points of piano teaching and the status quo of piano development of preschool children, this article analyzes the needs of the four types of users for the piano practice system, parents, teachers, students and principals, and studies special hardware, close connection with offline teaching scenes, easy-to-use abundant music score resources, and highly interactive piano preschool education online course platform.

## Figures and Tables

**Figure 1:** Cloud computing architecture.

**Figure 2:** Simulation diagram of a single access point table driving method.

**Figure 3:** Comparison diagram of single access point table driving method and ideal situation simulation.

**Figure 4:** System function module design.

**Figure 5:** System structure diagram.

**Table 1:** Parent table.

Field	Type of data	Remark
Id	int (ll)	Primary key id of the table
openid	varchar (64)	WeChat openid
Sign_up_time	datetime	Registration time
phone_number	varchar (20)	phone number
avatar	varchar (255)	Avatar URL
name	varchar (20)	Name

**Table 2:** Student table.

Field	Type of data	Remark
id	int (ll)	Primary key id of the table
name	varchar (16)	Name
gender	tinyint (4)	gender
background_year	varchar (255)	Background image URL
Learning_year	tinyint (4)	Year of piano
avatar	varchar (255)	Avatar URL
sign_up_time	datetime	Registration time
practice_duration	decimal (4, 2)	Total time of practice
practice_count	int (ll)	Total number of exercises
total_star	int (ll)	Total stars earned
family_id	int (ll)	Family id
is_available	tinyint (4)	Whether the current student has been deleted

**Table 3:** Parent_family_relationship table.

Field	Type of data	Remark
id	int (ll)	Primary key id of the table
parent_id	int (ll)	Parent's id
family_id	int (ll)	Family id
is_admin	tinyint (4)	Is the parent responsible for management
is_available	tinyint (4)	Whether the current parent-family relationship has been deleted
created_at	datetime	Creation time
relationship	tinyint (4)	Parents' relationship in the family

**Table 4:** Opern table.

Field	Type of data	Remark
id	int (ll)	Primary key id
illustration_path	varchar (255)	URL of the illustration
Opern_path	varchar (255)	The URL of the score
English_name	varchar (255)	English name of the score
name	varchar (16)	Score name
page_number	tinyint (4)	The page number of the score in the book
book_id	int (ll)	The id of the book where the score is located
created_at	datetime	Creation time
is_deleted	tinyint (4)	Whether to be deleted
Opern_data_path	varchar (255)	Data storage URL parsed from the score
is_one_hand	tinyint (4)	One-handed or two-handed

**Table 5:** Recording table.

Field	Type of data	Remark
Id	int (11)	Primary key id
created_at	datetime	Creation time
student_id	int (11)	Student id
demonstration_detail_id	int (11))	Specific demonstration id
homework_detail_id	int (11)	Specific job id
opern_name	varchar (16)	Score name
opern_id	int (11)	Score id
is_available	tinyint (4)	Whether to be deleted
audio_path	varchar (255)	Audio file address
algorithm_path	varchar (255)	Algorithm file address
playback_path	varchar (255)	Playback file address
recording_created_at	datetime	Record creation time
Star	mediumint (4)	Number of stars obtained
Size	decimal (4, 2)	The size of the recording file
Duration	decimal (4, 2)	Duration of recording
like_count	tinyint (4)	Likes
homework_id	int (11)	Big job id
parent_id	int (11)	Parent id
Type	tinyint (4)	Recording type
teacher_id	int (11)	Teacher id
Uuid	varchar (64)	Unique ID of iPad
Hand	tinyint (4)	Left-handed, right-handed or two-handed
is_long_shared	tinyint (4)	Long-term sharing
is_stick_top	tinyint (4)	Whether to top

## Data Availability

The data used to support the findings of this study are available from the corresponding author upon request.
